# The Relationship between Angiotensin–Neprilysin Treatment, Echocardiographic Parameters, and NT-proBNP Levels in HFpEF Patients with Acute Decompensated Heart Failure

This article has been retracted.

**DOI:** 10.1155/2022/4298644

**Published:** 2022-09-12

**Authors:** Xiaoliang Zhang, Song Yang, Zhonglin Xu

**Affiliations:** Department of Cardiovascular, The Ninth People's Hospital of Chongqing, No. 69, Jialing Village, Beibei District, Chongqing 400700, China

## Abstract

**Background:**

The valsartan-sacubitril therapy improved the outcomes of patients with acute decompensated heart failure (ADHF) of a reduced ejection fraction (HFrEF). In ADHF patients with preserved ejection fraction (HFpEF), it is not yet clear whether the same treatment regimen may be safely used to treat ADHF.

**Methods:**

For this study, HFpEF patients hospitalized due to ADHF were enrolled. Following hemodynamic stabilization, patients were randomized into two groups that were treated with enalapril or sacubitril-valsartan. In this trial, the primary efficacy outcomes were changes in echocardiographic parameters and NT-proBNP levels from baseline to 8 weeks treatment.

**Results:**

ARNI treatment resulted in a significant decrease in NT-proBNP levels and an increase in LVEF in patients with HFpEF. However, HFpEF patients that underwent ARNI treatment achieved better outcomes than did patients that underwent ACEI treatment.

**Conclusion:**

Sacubitril-valsartan treatment, which lowered NT-proBNP levels and improved cardiac function, was more effective in HFpEF patients with acute decompensated heart failure than enalapril.

## 1. Introduction

The worldwide public health concern of heart failure (HF) affects around 2% of people in developed countries [1, 2], resulting in symptoms associated with insufficient cardiac output [2, 3]. The three subtypes of heart failure are HF with reduced left ventricular ejection fraction (HFrEF) EF <40% (amended to ≤ 35%), HF with preserved LVEF (HFpEF) in patients with an EF greater than 50%, LV diastolic dysfunction, and evidence of structural heart disease (HFmrEF) in patients with an LVEF of 40-49%, diastolic dysfunction, increased BNP concentrations, and evidence of structural heart disease [4, 5]. The etiology and pathophysiological characteristics of HFpEF are complex and heterogeneous [6, 7], and even individuals specializing in HF may have difficulty accurately diagnosing this disease.

Succinylcholinesterase inhibitor (SCIE) therapy, which includes sacubitril and/or valsartan, has been shown to reduce symptoms and lower the odds of hospitalization owing to HF and cardiovascular death in chronic HFrEF patients relative to outcomes associated with the angiotensin-converting enzyme inhibitor (ACEI) enalapril, while is the gold standard approach to treating these patients [8]. Sacubitril-valsartan therapy was connected to substantial improvements in the severity of clinical symptoms among HFrEF patients as defined by hospitalization, LVE, NYHA NT-proBNP, and cardiovascular mortality in phase III randomized PARADIGM-HF study [9–11]. More recent studies have expanded on the findings of this trial and examined the establishment of multidrug regimens incorporating both neprilysin inhibitors and renin-angiotensin-aldosterone system (RAS) blockers [12].

The safety and efficacy of sacubitril-valsartan treatment were further compared to those of enalapril following hemodynamic stabilization in patients hospitalized with ADHF in the PIONEER-HF trial [13]. In this study, sacubitril-valsartan therapy was shown to be more effective than enalapril in reducing NT-proBNP concentrations in patients, whereas no differences in angioedema, hyperkalemia, worsening renal function, or symptomatic hypotension rates were evident among these groups [14, 15].

Up to now, sacubitril-valsartan does not have an indication in patients with HF with preserved ejection fraction (HFpEF) [16]. However, none of contemporary therapies was able to reduce HFpEF mortality. While sacubitril-valsartan was increasingly recognized as an efficacious treatment for HFrEF patients, whether it is similarly safe and effective in HFpEF patients undergoing hospitalization for acute decompensated HF remains to be established. The goal of this research was to compare the safety and efficacy of sacubitril-valsartan with enalapril in patients with heart failure, and treatment regimens in HFpEF patients hospitalized for ADHF. Our results suggest that sacubitril-valsartan treatment reduces NT-proBNP levels and improves cardiac function, and is more effective than enalapril in patients with HFpEF with acute decompensated heart failure. This provides new insights into the clinical treatment of HFpEF.

## 2. Material and Methods

### 2.1. Trial Design

The design for this trial has previously been published [14]. Study participants with ADHF were randomized, masked, and actively controlled to receive either enalapril or sacubitril-valsartan at the start of their stay in the hospital. The Chongqing Ninth People's Hospital's ethical committees have approved this study's protocol.

### 2.2. Patient Recruitment

The criteria for patient recruitment are as described previously [14]; in short, patients had to be at least 18 years old, have an LVEF of at least ≤ 50%, have BNP below ≤ 400 pg/mL, or N-terminal pro-B-type natriuretic peptide (NT-proBNP) values below ≤ 1600 pg/mL, and had been diagnosed with primary acute decompensated HF, which includes signs of fluid overload. Patients were enrolled while still hospitalized between 24 h and 10 days following initial hospital presentation. Patient randomization was only performed after hemodynamic stabilization, defined by an SBP ≥100 mmHg for at least 6 h without increases in i.v. diuretic doses and without the need for the administration of i.v. vasodilators over the past 6 h or i.v. inotropic agents over the past 24 h. Consent to treatment in the form of a written document was provided by every patient.

### 2.3. Trial Procedures

The criteria for patient recruitment were as described previously [14]; briefly, treatment with sacubitril-valsartan and enalapril (ACEI group) was randomized to patients. A fixed-dose combination of sacubitril-valsartan (either 24 mg of sacubitril with 26 mg of valsartan or 49 mg of sacubitril with 51 mg of valsartan as a fixed-dose combination) or enalapril (either 2.5 mg or 5 mg) was given twice daily to patients as an initial dosage. Blinding was achieved by providing all patients with a placebo resembling the other drugs. While patients in the enalapril group were administered enalapril and the placebo with their first dose, individuals treated with sacubitril-valsartan initially received two doses of placebos resembling both trial drugs such that a minimum washout period of 36 h prior to sacubitril-valsartan administration could be ensured, after which the appropriate trial drug and placebo were administered beginning with the third dose. A minimum of six hours of close observation followed the third dosage before patients were allowed to discharge. The sacubitril-valsartan dosage was tinkered with over the eight-week study period, with 97 and 103 mg twice-daily objectives for the two drugs. It was planned to have follow-up appointments in weeks one and two, and then every other week after that. On the morning of the eight-week follow-up appointment, the last medicine dosages were administered.

### 2.4. Trial Outcomes

This study's main finding was the time-averaged proportionate change in NT-proBNP levels between baseline and 4, 8, and 12 weeks after efficient treatment, as were echocardiographic parameters, including left ventricular end-diastolic dimension (LVEDD), left ventricular ejection fraction (LVEF), left ventricular end-systolic volume (LVESV), and left ventricular end-diastolic volume (LVEDV).

### 2.5. Statistical Analysis

All statistical analyses were performed using SPSS 21.0 (IL, USA). The Cox proportional-hazard models were used to compute hazard ratios and 95 percent confidence intervals (CIs), and log-rank test was used to compare the ACEI and ARNI treatment groups. It may not be feasible to replicate the conclusions reached from these intervals since the CIs for outcomes other than the main effectiveness outcome were not corrected for multiple comparisons. Treatment efficacy consistency was assessed in six pre-specified subgroups as well as six further exploratory subgroups. *p* < 0.05 was the significance threshold.

## 3. Results

### 3.1. The Impact of Sacubitril-Valsartan Treatment on Echocardiographic Parameters

Data from 127 patients who met the specified study inclusion criteria were gathered from the hospital information system registry of the Ninth People's Hospital of Chongqing between January 2018 and May 2019. Patient's characteristics at baseline are shown in Table 1. Patients in the ARNI and ACEI treatment groups exhibited a mean (±SD) age of 70.0 and 71.5 years, respectively (*p* =0.8563). The ARNI group consisted of 32 females (57.1%) and 24 males (42.9%) while the ACEI group consisted of 32 females (51.6%) and 30 males (48.4%). The mean SBP of patients in the ARNI and ACEI groups was 136.5 and 135.5 mmHg, respectively (*p* =0.7244), while corresponding DB*P* values were 76.5 and 77.0 mmHg (*p* =0.6832). In total, 8 (13.8%) and 10 (16.1%) of patients in the ARNI and ACEI groups had a history of smoking. No significant difference in the history of hypertension prior to HF was evident in these groups [42 (72.4%) vs 43 (69.4%), respectively, *p* =0.7126]. The history of diabetes mellitus was comparable between these patient cohorts [21 (36.2%) vs 26 (41.9%), respectively, *p* =0.5206]. Analysis of confounding factors showed that there were no differences in the baseline BP, age, gender, or medical history of the ACEI and ARNI patient groups.

Patients in the ARNI group had pre- and post-treatment LVEF values of 24.8 ± 5.7 and 44.3 ± 5.1, respectively, as shown in Tables 1 and 2, while for patients in the ACEI group, these respective values were 26.3 ± 6.1 and 36.3 ± 3.8. While significant increases in LVEF were evident in both groups, these increases were greater for HFpEF patients in the ARNI group. Pre- and post-treatment LVEDD values in the ARNI group were 61.3 ± 5.6 and 50.2 ± 4.6, respectively, while those in the ACEI group were 60.8 ± 6.7 and 54.6 ± 5.3. Pre- and post-treatment LVEDV values in the ARNI group were 176.4 ± 14.6 and 118.4 ± 17.6, while those in the ACEI group were 182.4 ± 15.4 and 146.3 ± 12.4, respectively. The LVESV values were 96.4 ± 11.7 before and after treatment in the ARNI group vs. 42.6 ± 14.7 after treatment, while those in the ACEI group were 98.7 ± 13.2 and 67.3 ± 16.7, respectively. The differences of LVEF, LVEDD, LVEDV, and LVESV values before and after treatment in ARNI group were significantly higher than those in ACEI group, suggesting that HFpEF patients that underwent ARNI treatment achieved better outcomes than did patients that underwent ACEI treatment (Table 2).

### 3.2. Changes in NT-proBNP Concentrations

To confirm the influence of ARNI and ACEI treatment on NT-proBNP expression, we firstly analyzed the baseline of NT-proBNP concentration in ARNI and ACEI pre-treatment groups. ELISA results showed that the NT-proBNP concentrations of the two groups did not vary (3284.62 ± 317.64 pg/mL vs. 3184.75 ± 486.37 pg/mL, Figure 1). In the two groups, after ARNI or ACEI treatment, the concentration of NT-proBNP was significantly higher than pre-treatment (Figure 2), and the concentration of NT-proBNP was dramatically lower in ARNI treatment group compared with ACEI treatment group (Figure 2).

## 4. Discussion

Up to now, sacubitril-valsartan does not have an indication in patients with HF with preserved ejection fraction (HFpEF) [16]. However, none of contemporary therapies is able to reduce HFpEF mortality. While sacubitril-valsartan is increasingly recognized as an efficacious treatment for HFrEF patients, whether it is similarly safe and effective in HFpEF patients undergoing hospitalization for acute decompensated HF remains to be established. NT-proBNP levels and echocardiographic parameters in patients with acute decompensated HFpEF were the focus of this study, which aims to compare the effects of sacubitril-valsartan and ACEI therapy. When follow-up was performed 8 weeks post-treatment, sacubitril-valsartan was found to be associated with significantly greater echocardiographic improvement and reduced NT-proBNP levels relative to those in HFpEF patients that underwent ACEI treatment. While LVEF improved significantly in both treatment groups, these improvements were more pronounced for individuals that were subject to ARNI treatment as compared to ACEI treatment. Several prior studies have reported similar LVEF improvement in patients diagnosed with HFrEF [17–20]. The PARAGON-HF study determined that sacubitril-valsartan treatment was associated with more pronounced absolute and relative benefit as compared to valsartan in HFpEF patients when this therapeutic regimen was initiated during the high-risk window following hospitalization, in line with the present study [21]. ARNI patients also exhibited significantly greater reductions in LVEDD, LVEDV, and LVESV as compared to the ACEI group. Similar left ventricular volume improvements have also been reported in other studies [22–25].

While NT-proBNP levels fell for patients in both treatment groups, these decreases were more pronounced in the ARNI group relative to the ACEI group. Patients with HFrEF have shown a decrease in NT-proBNP levels after treatment with sacubitril-valsartan [26–28]. Patients with acutely decompensated HF were not included in the PARADIGM-HF study since it focused on ambulatory patients with chronic HFrEF [29]. After randomization, 48-26%of patients in the sacubitril-valsartan and enalapril therapy groups had NT-proBNP levels reduced by more than >30% from baseline to one month after randomization, respectively [30]. Predischarge beginning of sacubitril-valsartan medication led in a 28 percent decline in NT-proBNP levels at discharge, according to a transitional trial of hospitalized acute decompensated HF patients [31]. In addition to LVEF, several other factors such as BMI, age, and creatinine clearance can also impact NT-proBNP levels [32]. In contrast to prior studies, HFpEF patients included herein underwent in-hospital randomization to undergo ARNI or ACEI treatment, while NT-proBNP levels were measured several weeks post-treatment. The results of this study, together with data from the PIONEER-HF and PARADIGM-HF trials, support the ability of sacubitril-valsartan treatment to rapidly decrease NT-proBNP levels irrespective of HF patient subtyping.

PIONEER-HF trial results provided an extended evidence base with respect to the utilization of sacubitril-valsartan in patients for whom little or no other data were available, including individuals with new-onset HF, individuals hospitalized for acute decompensated HF, individuals not receiving traditional RAS inhibitor therapy, or patients not receiving high dosages of HF medicines prescribed in accordance with current guidelines [33–35].

These findings support the safety of starting sacubitril-valsartan treatment in individuals with acute decompensated HFpEF. It was shown that sacubitril-valsartan was well tolerated throughout the in-hospital beginning phase of the PIONEER-HF trial and in a follow-up, open-label extension research.

## Figures and Tables

**Figure 1:** Pre-treatment NT-proBNP levels. Concentrations of NT-proBNP were compared at baseline between the ARNI and ACEI treatment groups. ns: no significance. ARNI group, *N* =58; ACEI group, *N* =62.

**Figure 2:** Pre- and post-treatment NT-proBNP levels. Concentrations of NT-proBNP were compared at baseline and at follow-up between the ACEI and ARNI treatment groups. ^∗^*p* < 0.05, ^∗∗^*p* < 0.01. ARNI group, *N* =58; ACEI group, *N* =62.

**Table 1:** General clinical data for patients in the ARNI and ACEI treatment groups.

Factors	ARNI	ACEI	*p*-value
	*N* =58	*N* =62	
Age	71.5 (66.0, 74.5)	70.0 (64.0, 72.0)	0.8563
Gender			
Male	24	30	0.5471
Female	32	32	
Smoking			
Yes	8	10	0.7203
No	50	52	
Hypertension			
Yes	42	43	0.7126
No	16	19	
Diabetes			
Yes	21	26	0.5206
No	37	36	
SBP (mmHg)	136.5 (128.5, 153)	135.5 (129.0, 155.0)	0.7244
DBP (mmHg)	76.5 (71.5, 92.0)	77.0 (72.5, 91.0)	0.6832
LVEF (%)	24.8 ± 5.7	26.3 ± 6.1	0.6274
LVEDD (mm)	61.3 ± 5.6	60.8 ± 6.7	0.6828
LVEDV (mL)	176.4 ± 14.6	182.4 ± 15.4	0.7144
LVESV (mL)	96.4 ± 11.7	98.7 ± 13.2	0.6632

**Table 2:** General clinical data for patients following ARNI and ACEI treatment.

Factors	ARNI treatment		ACEI treatment	
	Before	After	Before	After
LVEF (%)	24.8 ± 5.7	44.3 ± 5.1^∗∗^^,#^	26.3 ± 6.1	36.3 ± 3.8^∗^
LVEDD (mm)	61.3 ± 5.6	50.2 ± 4.6^∗∗^^,#^	60.8 ± 6.7	54.6 ± 5.3^∗^
LVEDV (mL)	176.4 ± 14.6	118.4 ± 17.6^∗∗^^,#^	182.4 ± 15.4	146.3 ± 12.4^∗^
LVESV (mL)	96.4 ± 11.7	42.6 ± 14.7^∗∗^^,#^	98.7 ± 13.2	67.3 ± 16.7^∗^

^∗^ *p* < 0.05 and ^∗∗^*p* < 0.01 compared with the before group; ^#^*p* < 0.05 compared with ACEI treatment.

## Data Availability

The data and study materials that support the findings of this study will be available to other researchers from the corresponding authors on reasonable request.
